The article "Comparison of Clinical Features and Inflammatory Markers between Kawasaki Disease Shock Syndrome and Kawasaki Disease without Shock: A Meta-Analysis" was retracted in 2023. Reasons: signs of a paper mill; suspected computer-generated content; unreliable results or conclusions; concerns about the data.

# Comparison of Clinical Features and Inflammatory Markers between Kawasaki Disease Shock Syndrome and Kawasaki Disease without Shock: A Meta-Analysis

**DOI:** 10.1155/2021/1486089

**Published:** 2021-12-20

**Authors:** Hui Zhang, Qin Zheng, Feng Li

**Affiliations:** ^1^Department of Pediatrics, The Central Hospital of Jiangjin, Jiangjin, Chongqing, China; ^2^Department of Pediatrics, Chongqing University Jiangjin Hospital, Jiangjin, Chongqing, China

## Abstract

Since the shock is not a common symptom of KD, it is often misdiagnosed at the beginning of the pathogenesis of KDSS. The language searched was only Chinese and English. Data from the articles were screened and extracted for meta-analysis using Stata16.0 software. A total of 9 cohort studies, including 1231 patients, were included in this meta-analysis. The results of meta-analysis showed that the age of the children in the KDSS group was higher than that in the KD group without shock, and the difference was statistically significant (SMD = 1.15, 95% CI (0.52, 1.78), *P* < 0.05); the CRP content in the KDSS group was higher than that in the KD group without shock, and the difference was statistically significant (SMD = 1.99, 95% CI (0.72, 3.26), *P* < 0.05); the albumin content in the KDSS group was lower than that in the KD group without shock, and the difference was statistically significant (SMD = −1.26, 95% CI (−1.85,−0.67), *P* < 0.05); the AST content in the KDSS group was higher than that in the KD group without shock, and the difference was statistically significant (WMD = 25.95, 95% CI (15.14, 36.75), *P* < 0.05); the difference had statistical significance (RR = 3.50, 95% CI (2.30, 5.32), *P* < 0.05); meta-analysis results of type of KD, fever duration, WBC count, ESR, ALT, and other outcome measures showed that there was no significant difference between KDSS and KD without shock (*P* > 0.05). Compared with KD without shock, children with KDSS are older and have a higher incidence of coronary artery disease, serum CRP, and AST, but albumin is lower than KD without shock. According to these characteristics, it may be helpful for the early identification of KDSS.

## 1. Introduction

Kawasaki disease (KD) is an acute, self-limiting, febrile disease involving the middle and small arteries throughout the body in children under five years of age [1–4]. The main manifestations of children are persistent fever, conjunctival congestion, acute noncervical lymphadenopathy, lip redness, rhagadia, and oedema of the extremities [5].

Based on the diagnosis of KD, some children may present with some less common clinical manifestations in the acute phase of the disease, such as hemodynamic instability, decreased blood pressure or even shock, systolic blood pressure persistently less than 20%, and more of the low normal systolic blood pressure in children of the same age, or clinical features combined with tissue hypoperfusion. In 1975, Kato et al. [6] reported a case of severe complications such as shock and heart failure in a 6-month-old child with KD. Since then, this critically ill KD with hemodynamic changes has been reported by successive investigators [7–11]. In 2009, Kanegaye et al. [12] first formally defined hemodynamically unstable Kawasaki disease as Kawasaki disease shock syndrome (KDSS), which accounts for approximately (1.9∼7.0)% of all KD. A study [13] has shown that children with Kawasaki disease admitted to the pediatric intensive care unit have severe and mostly atypical conditions, high resistance to intravenous gamma globulin, and rare organ damage and are easily misdiagnosed as sepsis or septic shock when macrophage activation syndrome or shock manifestations occur. Children with KDSS are often admitted to the pediatric intensive care unit with sepsis and septic shock [14]. Children may be diagnosed with incomplete/atypical KD even using the diagnostic criteria for KD [15]. The clinical manifestations of children with KDSS are usually accompanied by multisystem damage, involving the lungs, gastrointestinal tract, liver, and kidneys to varying degrees, and gastrointestinal symptoms are more prominent and rare, manifesting as vomiting, abdominal distension, abdominal pain, and diarrhoea [12, 16].

Children with KD are not promptly KDSS and may miss the optimal treatment time and aggravate the child's condition with some risk. Therefore, some investigators have compared the clinical features of children with KDSS and KD without shock to find characteristics that can help early identification of KDSS. Still, the results reported in various studies have not yet formed a consistent opinion. Therefore, this study aims to systematically evaluate the differences in the clinical features of KDSS and KD without shock by integrating the data of related studies and together provide guidance for the early diagnosis of KDSS in clinical practice.

## 2. Materials and Methods

### 2.1. Literature Search

PubMed, EMBASE, Cochrane Library, CNKI, VIP, Wangfang, and CBM were searched to collect relevant studies on comparing clinical features between KDSS and KD from inception to May 15, 2021, in Chinese and English only. Search terms are as follows: “Mucocutaneous Lymph Node Syndrome,” “Kawasaki disease,” “Kawasaki Syndrome,” “Lymph Node Syndrome, Mucocutaneous,” “Kawasaki disease shock syndrome”. English retrieval formula is as follows: ( (“Mucocutaneous Lymph Node Syndrome”[Mesh]) OR (((Kawasaki disease[Title/Abstract]) OR (Kawasaki Syndrome[Title/Abstract])) OR (Lymph Node Syndrome, Mucocutaneous[Title/Abstract]))) AND (Kawasaki disease shock syndrome[Title/Abstract]).

### 2.2. Inclusion and Exclusion Criteria

Inclusion criteria were as follows: (1) the study types selected for this meta-analysis were cohort study; (2) the experimental group of the study was KDSS patients; the control group was KD patients without shock; (3) the included studies needed to contain at least one of the following indicators: age, type of KD (CKD/IKD), fever duration, white blood cell (WBC) count, C-reactive protein (CRP), erythrocyte sedimentation rate (ES), albumin, alanine aminotransferase (ALT), aspartate aminotransferase (AST), coronary artery disease; (4) the included studies were all KDSS and KD patients without shock, and the diagnostic criteria of KDSS were as follows: on the basis of KD diagnosis, the children had hemodynamic instability, including systolic blood pressure persistently less than 20% of the low normal value of children of this age, or combined with clinical manifestations of tissue hypoperfusion, and required fluid resuscitation or vasoactive drugs to maintain normal blood pressure levels; and (5) the reported data in the complete literature of KDSS.

Exclusion criteria were as follows: (1) incomplete statistics or relevant data; (2) repeated publication of literature; (3) study subjects are not KDSS and KD without shock; and (4) conference, meta-analysis, and review of the literature.

### 2.3. Literature Screening and Data Extraction

The retrieved literature was initially screened by two investigators independently according to the inclusion and exclusion criteria and then cross-checked. The controversial literature was evaluated by the corresponding author (Feng Li) and then unified by discussion. Two investigators extracted the relevant information of the included literature, mainly including first author, publication year, publication country, sample size, age, type of KD (complete KD/incomplete KD, CKD/IKD), fever duration, WBC count, CRP, ESR, albumin, ALT, AST, and coronary artery disease.

### 2.4. Literature Quality Evaluation

The included studies were cohort controls. The quality assessment of the included articles was performed using the Newcastle–Ottawa scale (NOS), a quality evaluation tool specifically for case-control studies and cohort studies. The evaluation included three aspects: selection (four items), comparability (one item), and outcome (three items). Among them, the maximum score of each item of choice and outcome was 1, the total score of comparable items was 2, and the total score of scale evaluation results was 9. Scores (0∼4) were classified as low-quality articles, and (5∼9) as high-quality articles.

### 2.5. Statistical Methods

Meta-analysis of the data was performed using Stata16.0 software, enumeration data were expressed as relative risk (RR), measurement data were expressed as a weighted mean, standard deviation (WMD), or standardized difference (SMD), and interval estimation was described as 95% confidence interval (CI). Between-study heterogeneity was determined by the *χ*^2^ test combined with quantitative analysis of *I*^2^. If *P* > 0.01 and *I*^2^ < 50%, it was considered that between-study heterogeneity was acceptable, and the fixed-effect model was used for meta-analysis; if *P* < 0.01 and *I*^2^ > 50%, it was deemed that between-study heterogeneity was significant, and random-effect model was used for analysis. The Egger test judged the publication bias of the included studies, and *P* > 0.05 indicated no significant publication bias.

### 2.6. Ethics

The ethics were not available for the present study as the present study was a meta-analysis.

## 3. Results

### 3.1. Literature Search and Screening Results

In this meta-analysis, 585 relevant pieces of literature were obtained through preliminary retrieval, of which 412 remained after excluding repeated literature, 37 remained after excluding irrelevant study through the reading title, and nine remained after excluding abstract, animal study, and review through reading full text [12, 16–23], all of which were cohort studies, including 7 English articles and 2 Chinese articles, involving 1231 patients.  Figure 1 is the flowchart of literature search and screening.

### 3.2. Basic Characteristics and Quality Assessment of Included Literature

Nine articles were included in this meta-analysis, and Table 1 is the basic characteristics of the studies. The quality of the included studies was evaluated, and all articles had NOS scale scores ≥ 5, suggesting that the overall quality of the included articles was high.

### 3.3. Meta-Analysis Results

#### 3.3.1. Meta-Analysis on the Age of Children

Nine studies [12, 16–23] reported the age of the children, and the heterogeneity of the included studies was tested (*I*^2^ = 90.0%, *P* < 0.001), indicating that there was high heterogeneity among the included studies, and the effect size was combined using a random-effects model, and the results showed that (SMD = 1.15, 95% CI (0.52, 1.78)), which suggested that the age of the children in the KDSS group was higher than that in the KD group without shock, and the difference was statistically significant (*P* < 0.05).  Figure 2 is the forest plot of age comparison of KD patients without shock in KDSS.

#### 3.3.2. Meta-Analysis of Fever Duration

Fever duration was reported in six studies [16, 18, 21–23]. The heterogeneity test was performed for the included studies (*I*^2^ = 83.2%, *P* < 0.001), indicating high heterogeneity among the included studies. The random-effects model was used to combine the effect size. The results showed (WMD = 1.33, 95% CI (−0.18, 2.83)), suggesting that there was no significant difference in fever duration between KD patients without shock in the KDSS KD group (*P* > 0.05).  Figure 3 is the forest map of fever duration comparison in KD patients without shock in KDSS.

#### 3.3.3. Meta-Analysis of WBC Count

There were seven studies [12, 16, 19, 22, 23] that reported WBC count. The heterogeneity test was performed for the included studies (*I*^2^ = 82.1%, *P* < 0.001), indicating high heterogeneity among the included studies. The random-effects model was used to combine the effect size. The results showed (WMD = 2.37, 95% CI (−0.42, 5.16)), suggesting that there was no significant difference in WBC count between the KDSS and KD group patients (*P* > 0.05).  Figure 4 is the forest plot for comparison of WBC counts in KDSS patients without shock KD.

#### 3.3.4. Meta-Analysis of CRP

CRP was reported in seven studies [12, 16, 19, 22, 23]. The heterogeneity of the included studies was tested (*I*^2^ = 96.5%, *P* < 0.001), indicating that there was high heterogeneity among the included studies. The effect size was combined using a random-effects model. The results showed that (SMD = 1.99, 95% CI (0.72, 3.26)), which suggested that the CRP content in patients in the KDSS group was higher than that in the KD group without shock, and the difference was statistically significant (*P* < 0.05).  Figure 5 is the forest plot of CRP comparison in KD patients without shock in KDSS.

#### 3.3.5. Meta-Analysis of ESR

ESR was reported in five studies [12, 16, 18, 23]. A heterogeneity test was performed for the included studies (*I*^2^ = 90.7%, *P* < 0.001), indicating high heterogeneity among the included studies. The random-effects model was used to combine the effect size. The results showed (WMD = 1.15, 95% CI (−19.88, 22.18)), suggesting that there was no significant difference in ESR between KD patients without shock in KDSS (*P* > 0.05).  Figure 6 is the forest plot of ESR comparison in KD patients without shock in KDSS.

#### 3.3.6. Meta-Analysis of Albumin

Albumin was reported in six studies [16, 19, 22, 23], and the heterogeneity of the included studies was tested (*I*^2^ = 83.3%, *P* < 0.001), indicating that there was high heterogeneity among the included studies, and the effect size was combined using a random-effects model, and the results showed that (SMD = −1.26, 95% CI (−1.85, −0.67)), which suggested that the albumin content in patients in the KDSS group was lower than that in the KD group without shock. The difference was statistically significant (*P* < 0.05).  Figure 7 is the forest plot of albumin comparison in KD patients without shock in KDSS.

#### 3.3.7. Meta-Analysis of ALT

ALT was reported in four studies [17, 19, 22]. A heterogeneity test was performed for the included studies (*I*^2^ = 94.2%, *P* < 0.001), indicating high heterogeneity among the included studies. The random-effects model was used to combine the effect size. The results showed (WMD = 89.02, 95% CI (−15.70, 193.74)), suggesting that there was no significant difference in ALT content between KDSS and KD patients without shock (*P* > 0.05) Figure 8 is the forest plot of ALT comparison in KD patients without shock in KDSS.

#### 3.3.8. Meta-Analysis of AST

AST was reported in four studies [17, 19, 22]. The heterogeneity of the included studies was tested (*I*^2^ = 0.0%, *P*=0.761), indicating that there was no heterogeneity among the included studies. The fixed-effect model was used to combine the effect size. The results showed that (WMD = 25.95, 95% CI (15.14, 36.75)), suggesting that the AST content in the KDSS group was higher than that in the KD group without shock, and the difference had statistical significance (*P* < 0.05).  Figure 9 is the forest plot of AST comparison in KD patients without shock in KDSS.

#### 3.3.9. Meta-Analysis of Type of KD (CKD/IKD)

There were seven studies [16–22] that reported the type of KD. The heterogeneity of the included studies was tested (*I*^2^ = 46.6%, *P*=0.081), indicating that there was moderate heterogeneity among the included studies. The fixed-effect model was used to combine the effect size. The results showed (RR = 1.05, 95% CI (0.88, 1.24)), suggesting that there was no significant difference in the incidence rate of CKD and IKD (*P* > 0.05).  Figure 10 is the forest plot of the type of KD comparison in KDSS patients without shock KD group.

#### 3.3.10. Meta-Analysis of Coronary Artery Disease

Coronary artery disease was reported in five studies [16, 19, 22]. The heterogeneity of the included studies was tested (*I*^2^ = 34.1%, *P*=0.194), indicating that there was moderate heterogeneity among the included studies. The effect size was combined using a fixed-effect model. The results showed that (RR = 3.50, 95% CI (2.30, 5.32)), which suggested that the incidence of coronary artery disease in patients in the KDSS group was higher than that in the KD group without shock. The difference was statistically significant (*P* < 0.05).  Figure 11 is the forest map of coronary artery disease comparison in KD patients without shock in KDSS.

### 3.4. Sensitivity Analyses

Due to the significant heterogeneity of the included literature for outcome measures such as age, fever duration, WBC count, CRP, ESR, albumin, and ALT, sensitivity analysis is required. In the sensitivity analysis of outcome measures such as fever duration, WBC count, CRP, and ALT, no primary source of increased heterogeneity was found by the one-by-one elimination method. In the sensitivity analysis of age, it was found that the study by Huixian Qiu et al. [19] was the primary source of increased heterogeneity by the one-by-one elimination method. After excluding this article, the obtained results showed that the age of children in the KDSS group was higher than that in the KD group without shock. The difference was statistically significant (*P* < 0.05), indicating that the results of this study were relatively stable and reliable. In the sensitivity analysis of albumin, it was found that the study by Weibin Li et al. [23] was the primary source of increased heterogeneity. After excluding this article, it was shown that the patients in the KDSS group had lower albumin than those in the KD group without shock. The difference was statistically significant (*P* < 0.05), indicating that the results of this study were unstable. In the sensitivity analysis of ESR, it was found that the study by Yandie Li et al. [18] was the primary source of increased heterogeneity. The results obtained after excluding this article showed no significant difference in ESR between KDSS patients without shock and KD patients without shock (*P* > 0.05), indicating that the results of this study were relatively stable and reliable.

### 3.5. Publication Bias

Since only nine pieces of literature were included in this study, the publication bias could not be effectively assessed through a funnel plot. Egger's test was used to evaluate the publication bias of age, type of KD (CKD/IKD), fever duration, WBC count, CRP, ESR, albumin, ALT, AST, coronary artery disease, and other outcome measures. The results showed that age (*P*=0.073), type of KD (*P*=0.273), fever duration (*P*=0.069), WBC count (*P*=0.019), CRP (*P*=0.208), ESR (*P*=0.364), albumin (*P*=0.387), ALT (*P*=0.116), AST (*P*=0.774), and coronary artery disease (*P*=0.260) suggested that the studies only included in WBC outcome measures had publication bias (*P* < 0.05), and the other outcome measures had no publication bias (*P* > 0.05).

## 4. Discussion

In our study, we found that the age of onset of children with KDSS was older than that of children with KD without shock, the contents of serum CRP and AST in children with KDSS were significantly higher than those of children with KD without shock, and the incidence of coronary artery disease was also higher than that of children with KD without shock. Among the ten outcome measures studied, only the contents of serum albumin in children with KDSS were lower than those of children with KD without shock, and the results of the other five outcome measures (type of KD, fever duration, WBC count, ESR, and ALT) showed no significant difference between the KDSS group without shock and the KD group without shock. According to the characteristics of older age, increased serum CRP and AST levels and decreased serum albumin content in children may be helpful for early identification of KDSS as an effective differential diagnostic indicator of KDSS and KD without shock.

There are an increasing number of studies on KDSS and a growing number of reports of related diseases. In two survey studies of KD in Taiwan, it was found that the incidence of KDSS in children with KD ranged from 1.45% to 1.51%, with the highest incidence in children in the age group of 8∼9 years [24, 25]. Some regional survey reports in mainland China showed that the overall incidence of KDSS ranged from 1.16% to 1.23%, with older children being rare [18]. Surveys in Western countries have shown a higher incidence of 5% to 12.3% than in Asian regions. The age distribution is irregular in children younger than six months or older, who have a greater median age than KD children without shock [20, 26]. In the present study, our meta-analysis also showed that children with KDSS were older than children with KD without shock, consistent with the results of these investigative studies.

Persistent fever is a common clinical manifestation in children with KD, and in our study analysis, the fever duration was not higher in KDSS children than in KD children without shock. In addition, the difference between the diagnostic yield of complete KD and that of incomplete KD in patients with KDSS was also not significantly different. Therefore, it does not seem to be helpful in the differential diagnosis of KDSS and KD without shock in terms of body temperature and the type of KD.

At present, the pathogenesis of KDSS is still unclear, and it is speculated that it may be related to a combination of mechanisms such as capillary leakage caused by intense systemic vasculitis, immune dysregulation, and systemic inflammatory response caused by infection, myocardial dysfunction, and abnormal cytokine regulation [27, 28]. The type of shock in KDSS can be characterized by distributive shock dominated by capillary leakage, cardiogenic shock dominated by myocardial dysfunction, or both shocks. For the diagnosis of KD, inflammatory parameters such as CRP, ESR, and WBA count are necessary, and theoretically, vasculitis is more severe in children with KDSS. Therefore, the above parameters may be more significantly increased in KDSS. But our study analyzed the difference of serum CRP and WBC count in patients and only found that CRP was significantly different. As an acute-phase protein, CRP may reflect that KDSS patients are in the acute-phase response phase. The nondifferential nature of WBC counts reflects that the onset of KDSS patients may be more due to noninfectious factors. Subsequent pathogenesis studies may pay more attention to noninfectious factors. Li Y et al. [18] showed that the levels of peripheral blood cytokines interleukin-6 (IL-6), interleukin-10 (IL-10), tumour necrosis factor-*α* (TNF-*α*), and interferon-*γ* (INF-*γ*) were significantly higher in the KDSS group than in the KD group without shock. When IL-6 > 66.7 pg/mL, IL-10 > 20.85 pg/mL, and IFN-*γ* > 8.35 pg/mL, the sensitivity and specificity for distinguishing KDSS from KD without shock were 85.2% and 62.8%, and 66.7% and 83.7%, respectively. Few relevant studies focus on the levels of cellular inflammatory factors, and the search for cutoff values with differential significance from cytokine levels requires controlled studies with large samples. KDSS patients can also present with a range of abnormal blood biochemical tests. Our study found decreased serum albumin and increased AST content, closely related to the high levels of cytokines. Albumin acts as a negative protein of the inflammatory response, and high levels of cellular inflammatory factors inhibit the formation or secretion of albumin [29, 30]. The increase in AST also reflects that KDSS patients are prone to liver damage [16].

Cytokines have a role in assisting in differentiating KDSS from KD without shock but are difficult in determining toxic shock or septic shock. KDSS is often treated as toxic shock or septic shock at the beginning of the disease, and pediatricians consider the diagnosis of KDSS when the initial treatment is insufficient or coronary artery changes are found by echocardiography [15, 31, 32]. KDSS is very similar to septic shock in clinical features and inflammatory parameters and is difficult to differentiate. The development of septic shock is dominated by microcirculatory dysfunction, and tissue hypoperfusion is difficult to assess with systemic hemodynamics. When blood pressure decreases in septic shock, it indicates that the patient has entered decompensation, is in critical condition, is rapidly associated with multiple organ failure, and has a high mortality rate. Rescue of septic shock in addition to the use of vasoactive drugs, normal saline volume expansion, or albumin must be given to correct hypotension, and hormonal therapy has some benefit but is not the first. Children with KDSS generally do not experience coma and multiple organ failure and rarely develop coagulation abnormalities and thrombocytopenia, and blood pressure is easily controlled after using vasoactive drugs. The dose of vasoactive drugs does not need to be very large; the condition can be relieved after KDSS treatment with hormones and immunoglobulins. At the same time, the septic shock has a poor therapeutic effect on hormones and immunoglobulins [16]. Most of the KDSS have different degrees of diagnostic delay at the initial admission. Given the overlap of KDSS with toxic shock and septic shock in symptoms, it is difficult to differentiate the three from symptoms alone. Echocardiography shows more myocarditis (cardiomegaly and reduced cardiac function), abnormal coronary artery lesions, and valvular lesions, while toxic shock and septic shock often present with high-output and low-resistance shock while myocardial depression and valvular lesions are rare, so echocardiography may be a sensitive tool for early differentiation. Repeated echocardiographic examinations were performed to detect changes in a coronary artery, myocardial, and valve function on time. This study also confirmed that children with KDSS are more likely to develop coronary artery abnormalities, and the changes can be used as an auxiliary diagnosis of KDSS.

In this study, we analyzed the differences in clinical features and inflammatory parameters between KDSS and KD without shock, compared KDSS and KD without shock for the first time, and found that characteristics such as age, serum CRP, AST content, and serum albumin content may be helpful for early identification of KDSS. The conclusion obtained in this study is more persuasive than the results reported in single literature and can provide some guiding value for clinical diagnosis. However, this study also had some limitations. First, because the included literature was cohort studies, the quality of this original literature was not as good as that of randomized controlled trials; second, due to the limited number of serological indicators concerned in this study, the detailed analysis of each serum indicator could not be conducted. Although the conclusion of this study only found some characteristics with differences, no specific diagnostic indicators were found, and the diagnostic cutoff values of the corresponding indicators were not found.

## 5. Conclusion

According to the data of the existing literature, children with KDSS were older. They had a higher incidence of coronary artery disease, serum CRP, and AST but lower albumin than KD children without shock. As pediatricians, KDSS should be fully recognized, vigilance for diagnosis should be improved, and the possibility of KDSS should be timely identified in cases of fever of unknown origin with shock and concurrent multiple organ damage. Given that the aetiology and pathogenesis of Kawasaki disease are still not clear, subsequent studies can continue to investigate the aetiology and pathogenesis of KDSS and then find specific diagnostic indicators from the aetiology and pathogenesis possible.

## Figures and Tables

**Figure 1:** Flowchart of literature search and screening.

**Figure 2:** Forest plot of age comparison of KD patients without shock in KDSS.

**Figure 3:** Forest map of fever duration comparison in KD patients without shock in KDSS.

**Figure 4:** Forest plot for comparison of WBC counts in KDSS patients without shock KD.

**Figure 5:** Forest plot of CRP comparison in KD patients without shock in KDSS.

**Figure 6:** Forest plot of ESR comparison in KD patients without shock in KDSS.

**Figure 7:** Forest plot of albumin comparison in KD patients without shock in KDSS.

**Figure 8:** Forest plot of ALT comparison in KD patients without shock in KDSS.

**Figure 9:** Forest plot of AST comparison in KD patients without shock in KDSS.

**Figure 10:** Forest plot of type of KD comparison in KDSS patients without shock KD group.

**Figure 11:** Forest map of coronary artery disease comparison in KD patients without shock in KDSS.

**Table 1:** Basic characteristics and quality evaluation results of the included literature.

Study	Gender (M/F)		Age		Sample sizes		Type of KD (CKD/IKD)		Fever duration (d)		NOS scores
	KDSS	KD without shock	KDSS	KD without shock	KDSS	KD without shock	KDSS	KD without shock	KDSS	KD without shock	
Chen et al. [17]	11/10	13/11	4.9 ± 2.8 y	2.7 ± 1.9 y	21	24	16/5	16/8	6.7 ± 2.4	5.3 ± 0.6	7
Ma et al. [18]	17/10	19/24	43.41 ± 31.42 m	28.81 ± 21.51 m	27	43	8/19	2/41	10.63 ± 5.12	6.98 ± 2.45	6
Li et al. [19]	14/3	45/23	49.6∼90.0 m	14.2∼45.0 m	17	68	15/2	54/14	4∼5	NA	6
Qui et al. [20]	8/3	126/77	3∼120 m	2∼186 m	11	203	4/7	145/58	NA	NA	6
Gao et al. [16]	3/6	16/11	3.2 ± 3.3 y	2.0 ± 1.8	9	27	7/2	17/10	9.0 ± 3.1	7.1 ± 2.3	5
Gámez-González et al. [21]	6/7	53/38	0.5∼10.6 y	0.2∼8.4 y	13	91	6/5	61/27	8–23	3–29	6
Yang et al. [12]	4/9	104/70	2.2∼5.9 y	0.9∼3.9 y	13	174	NA	NA	NA	NA	7
Park et al. [22]	8/3	48/13	4.41 ± 3.62 y	3.17 ± 1.74 y	11	61	9/2	51/10	6.45 ± 2.27	6.39 ± 1.50	7
Shan et al. [23]	13/10	257/138	44 ± 23 m	22 ± 33 m	23	395	NA	NA	7.00 ± 2.00	6.00 ± 2.00	5

M： male; F： female; IKD: incomplete KD; CKD: complete KD; NA: not available; d: days; m: months; y: years; ①： age; ②: type of KD (CKD/IKD); ③: fever duration; ④: WBC count; ⑤: CRP; ⑥: ESR; ⑦: albumin; ⑧: alanine aminotransferase (ALT); ⑨: aspartate aminotransferase （AST）; ⑩ coronary artery disease.

## Data Availability

The simulation experiment data used to support the findings of this study are available from the corresponding author upon request.
